RETRACTED

# MicroRNA-641 Inhibits Endometrial Cancer Progression via Targeting AP1G1

**DOI:** 10.1155/2022/7918596

**Published:** 2022-09-30

**Authors:** Yanfen Dong, He Yang, Handan Hua

**Affiliations:** ^1^Department of Laboratory, The Affiliated Changzhou Second People's Hospital of Nanjing Medical University, Changzhou 213003, China; ^2^Department of Gynecology, The Affiliated Changzhou Second People's Hospital of Nanjing Medical University, Changzhou 213003, China

## Abstract

MicroRNA-641 (miR-641) was significantly decreased in various cancers, but its roles in endometrial cancer (EC) remain unclear. We explored the influences of miR-641 on the EC cells. In our study, the miR-641 expression was reduced in EC cells. Overexpression of miR-641 inhibited viability and proliferation of HEC-1A and HECCL-1 cells by CCK-8 and colony formation assays. Additionally, flow cytometry revealed that overexpression of miR-641 could remarkably promote apoptosis and arrest the cell cycle at the G1 phase of HEC-1A and HECCL-1 cells. Besides, forced expression of miR-641 suppressed the migration and invasion of HEC-1A and HECCL-1 cells as evidenced by wound healing and transwell assay. Moreover, AP1G1 was confirmed as a target gene of miR-641 by StarBase prediction and DLR assay and their expressions were negatively correlated. Overexpression of AP1G1 neutralized the roles of miR-641 mimic on the viability, proliferation, apoptosis, and migration of HEC-1A and HECCL-1 cells. Our findings illustrated that miR-641 was reduced in the EC cells and AP1G1 antagonized the miR-641 mimic-induced inhibition of the EC progression *in vitro*. Therefore, miR-641 may emerge as an effective molecule for EC treatment.

## 1. Introduction

Endometrial cancer (EC) is a reproductive system tumor in females and ranks fourth in developed countries. Furthermore, in developing countries, the incidence rate of EC is also in the seventh place in female tumors. EC often occurs in postmenopausal women, but in recent years, clinical research shows that EC has a significant trend in youth [1, 2]. After standardized treatment, the 5-year survival rate rises year by year. The late prognosis of late, poorly differentiated EC or special types is an important factor leading to death. Therefore, to improve the prognosis of EC, it is necessary to investigate the pathogenesis and effective targets of EC [3].

At present, most studies show that EC is related to obesity, hypertension, diabetes, or long-term exposure to estrogen without progesterone antagonists [4–6]. However, at the molecular level, the mechanism of EC is not clear and the abnormal gene regulation, such as the imbalance of oncogenes, tumor suppressor genes, and polymorphism, cannot fully explain the pathogenesis of EC [7, 8]. It has been shown that microRNAs (miRNAs), noncoding single strand small molecules with 19–25 nucleotides in length could mediate the progression of EC [9, 10]. For example, miR-135a was upregulated in the EC cells and the overexpression of miR-135a could increase proliferation and metastasis while inducing chemoresistance of the EC cells [11]. Additionally, miR-214-3p was impoverished in EC tissues and cell lines. Upregulation of miR-214-3p suppressed metastasis of the EC cells through inhibition of EMT via targeting TWIST1 [12]. Therefore, miRNAs may be effective targets for EC therapy.

miRNA-641 (miR-641) exhibited an essential role in lung cancer, cervical carcinoma, and glioblastoma [13–15]. However, its mechanism in the EC cells remain unknown. Herein, we evaluated miR-641 expression in the EC cells, the detailed role, and possible mechanisms were determined.

RETRACTED

## 2. Materials and Methods

### 2.1. Cells

HEC-251 and EC cell lines HEC-1A, RF952, HECCL-1, and BMDC1 were bought from the Chinese Academy of Science and incubated with DMEM (Gibco, USA) plus 10% FBS (Gibco, USA) and antibiotics in a humidified 5% CO_2_ incubator at 37°C.

### 2.2. Transfection

miR-641 mimic/mimic NC and specific siRNAs against AP1G1, the pcDNA3.1 vector targeting AP1G1 and the empty vector (Genechem, China) were transfected into the EC cell lines via Lipofectamine 3000 (Thermo Fisher, USA).

### 2.3. CCK-8 Assay

The transfected HEC-1A and HECCL-1 cells (1 × 10^4^ cells/well) were kept in 96-well plates and incubated for indicated times. The viability was tested by a CCK-8 kit (Beyotime, China). OD was recorded at 450 nm by Tecan Infinite M200 (LabX, Switzerland).

### 2.4. Colony Formation Assay

HEC-1A and HECCL-1 cells (1 × 10^3^/well) were cultured in 6-well plates with a refreshing medium every 3 days for 14 days. Then, the cells were stained with 10% crystal violet to determine the proliferative ability.

### 2.5. Flow Cytometry

1 × 10^6^/mL transfected HEC-1A and HECCL-1 cells were fixed with 70% ethanol at 4°C overnight. After washing, 100 *μ*L of RNase A was administrated for 30 min at 37°C and 400 *μ*L of PI dye solution and was applied and incubated for 0.5 h at 4°C. The cell cycle was checked using a flow cytometer (BD, USA).

The transfected HEC-1A and HECCL-1 cells were harvested and resuspended. Then, the cells were treated with Annexin V-FITC (5 *μ*L) and PI (10 *μ*L). The apoptosis was measured.

### 2.6. Wound Healing Assay

HEC-1A and HECCL-1 cells (5 × 10^5^ cells/well) were kept in 6-well plates. After the confluence reached 80%, a 10 *μ*L pipette tip wound of the monolayer and the cells were cultured continuously. The cells were photographed at 48 h with inverted microscopy (Tokyo, Japan).

RETRACTED

### 2.7. Transwell Assay

The transfected HEC-1A and HECCL-1 (1 × 10^6^ cells/well) were seeded into the upper chamber of the transwell equipment (Corning, USA) with serum-free DMEM medium. The lower chamber had DMEM with 20% FBS. To check the invasion of cells, Matrigel (Becton-Dickinson, USA) was transferred to the upper chambers. After 48 h, the cells were stained with 0.5% crystal violet and observed with inverted microscopy (Tokyo, Japan).

### 2.8. Dual-Luciferase Reporter (DLR) Assay

Wild type and mutant AP1G1 3'-UTR vectors were synthesized by subcloning AP1G1 3'-UTR and mutant 3'-UTR sequences into the plasmids (Promega, USA). Then, HEC-1A and HECCL-1 were co-transfected with reporter vectors (80 ng) and miR-641 mimic/NC mimic using Lipofectamine 3000 (Thermo Fisher, USA). After 48 h, luciferase activities were recorded.

### 2.9. RT-qPCR Assay

RNA was separated by Trizol (Invitrogen, USA) and synthesized to cDNA with a TaqMan Reverse Transcription Kit (AB, USA). RT-qPCR was implemented using ABI 7300 (AB, USA) with a SYBR Green PCR Kit (Qiagen, USA). Relative expression was evaluated by the 2^−ΔΔCt^ method. The primers were as follows: miR-641 forward, 5′-TTATACTCTCACCATTTGGATC-3′, reverse, 5′-TGACAAGATTTTACATCAAG AA-3′. U6 forward, 5′-CTCGCTTCGGCAGCACATA-3′, reverse, 5′-AACGCTTCACGAATTT GCGT-3′.

### 2.10. Western Blot

Protein was isolated and quantified via a BCA kit (Beyotime, China), separated through 12% SDS-PAGE, shifted into PVDF membranes (Millipore, USA) and sealed with 5% non-fat milk. Then, the samples were treated with the primary antibodies, probed with a HRP-conjugated secondary antibody (1 : 2,000, ab6728), observed with an ECL kit (Millipore, USA) and analyzed via Image J. The primary antibodies were as follows: anti-Cyclin D1 (1 : 1, 000, ab16663), anti-CDK2 (1 : 1000, ab32147), anti-PCNA (1 : 1000, ab92552), anti-COX2 (1 : 1000, ab15191), anti-MMP-2 (1 : 1000, ab97779), anti-MMP-9 (1 : 1000, ab38898), anti-APP1G1 (1 : 1000, ab167153), and anti-*β*-actin (1 : 2, 000, ab8227) (Abcam, USA).

### 2.11. Statistical Analysis

Data were processed by the GraphPad Prism 5.0 and exhibited as the mean ± SD. ANOVA followed by Tukey's POC host calculated the differences between the groups. *P* < 0.05 indicated a statistical significance.

## 3. Results

### 3.1. miR-641 Is Downregulated in the EC Cells and miR-641 Mimics Suppresses Viability and Proliferation of the EC Cells

First, RT-qPCR was employed to evaluate the miR-641 expression in HEC-251 and the EC cell lines HEC-1A, RF952, HECCL-1, and BMDC1.  Figure 1(a) demonstrates that miR-641 was lessened in the EC cells compared with HEC-251 cells, especially in HEC-1A and HECCL-1 cells. Moreover, miR-641 mimic and miR-641 mimic NC were transfected into HEC-1A and HECCL-1 cells and the efficiency was evaluated by RT-qPCR assay.  Figure 1(b) reports that miR-641 in HEC-1A and HECCL-1 cells transfected with miR-641 mimic was increased relatively to the miR-641 mimic NC group. In addition, Figure 1(c) displays that overexpression of miR-641 diminished the viabilities of HEC-1A and HECCL-1 cells. Furthermore, the proliferation of HEC-1A and HECCL-1 cells was detected and miR-641 mimic inhibited the proliferation of HEC-1A and HECCL-1 cells relative to miR-641 mimic NC (Figure 1(d)). These suggested that the EC cells has a low level of miR-641 and its overexpression inhibited cell viability and proliferation.

RETRACTED

### 3.2. Upregulation of miR-641 Accelerates Apoptosis and Induces the G1 Phase Arrest of the EC Cells

Flow cytometry was performed and the data showed that the miR-641 mimic caused the apoptosis of HEC-1A and HECCL-1 cells compared to the miR-641 mimic NC group (Figure 2(a)). Additionally, it was found that miR-641 mimic triggered cell cycle arrest in the G1 phase of HEC-1A and HECCL-1 cells compared to the miR-641 mimic NC group (Figure 2(b)). Furthermore, the results of the Western blot in Figure 2(c) indicate that upregulation of miR-641 inhibited the protein levels of Cyclin D1 and CDK2, whereas the P21 expression was promoted in HEC-1A and HECCL-1 cells. These evinced that cell apoptosis and cell cycle arrest in the G1 phase are triggered by upregulation of miR-641.

### 3.3. Upregulation of miR-641 Retards Metastasis of the EC Cells

Wound healing and transwell assays determined the role of miR-641 in the EC cell migration and invasion.  Figure 3(a) illustrates that the miR-641 mimic suppressed the migration of HEC-1A and HECCL-1 cells compared to the miR-641 mimic NC group. In addition, Figure 3(b) reports that miR-641 mimic reduced the metastasis of both the cell lines. Furthermore, the levels of metastasis-associated proteins were checked and the data in Figure 3(c) reveal that the levels of Cox-2, MMP-2, and MMP-9 were reduced in the cells transfected with miR-641 mimic. These summarized that metastasis of the EC cells is caused by the upregulation of miR-641.

### 3.4. AP1G1 Is Sponged by miR-641 in the EC Cells

miRNAs function as oncogenes or antioncogenes via sponging downstream target genes. In Figure 4(a), using StarBase, AP1G1 was predicted as a possible target of miR-641 and it was proved to manage the development of colon cancer and breast cancer [16–18]. Furthermore, it was detected by DLR assay that miR-641 weakened the luciferase activity of 3'UTR of AP1G1 mRNA, whereas the suppressive effect was terminated by the mutation on the binding sites (Figure 4(b)). Moreover, the AP1G1 expression in the miR-641 mimic-transfected HEC-1A and HECCL-1 cells were assessed. In Figures 4(c) and 4(d), the levels of AP1G1 were dropped in miR-641 mimic-transfected cells. These results proved that AP1G1 was sponged by miR-641 in EC.

RETRACTED

### 3.5. AP1G1 Affects the Roles of miR-641 on the EC Cells

The cells were infected with Lv-AP1G1, and the efficacy was determined by RT-qPCR assay and the data are given in Figure 5(a). Functionally, the result of the CCK-8 assay emerged that overexpression of AP1G1 eliminated the prominent reduction in proliferation of HEC-1A and HECCL-1 cells transfected with miR-641 mimic (Figure 5(b)). Colony formation assay also unveiled that the overexpression of AP1G1 altered the impaired proliferative ability of cells transfected with miR-641 mimic (Figure 5(c)). Correspondingly, the promotive impacts of miR-641 mimic on cell apoptosis cells were ameliorated by AP1G1 overexpression (Figure 5(d)). Moreover, the transwell assay manifested that overexpression of AP1G1 compensated inhibitory influence of miR-641 mimic on the metastasis of both the cell lines (Figure 5(e)). These data summarized that AP1G1 took part in the function of miR-641 in EC.

## 4. Discussion

EC is a heterogeneous tumor derived from endometrium with different histological types and is a common malignancy with a 53% survival rate within 5 years [19]. The mortality rate of EC has gradually risen and tends to be younger [20]. Hence, the development of new biomarkers has become the main means of diagnosis and therapy of EC.

miRNAs, as a group of short sequence RNAs, do not encode proteins with a length of about 19–25 nt and are widely distributed in eukaryotes. In addition, their synthesis is an extremely complex biological process, mainly in the cytoplasm and nucleus [21]. miRNAs can regulate cell survival, differentiation, and response to the external environment through degrading target gene miRNAs or inhibiting the expression of regulatory genes in the translation process via the incomplete complementary pairing of their “seed” sequence with the 3'-UTR region of target gene miRNAs [22]. MicroRNAs control EC at different stages of development, and their abnormal expression in tumors plays a dual role in promoting or inhibiting cancer. For example, miR-125b was upregulated in EC and the silence of miR-125b retard the proliferation and enhance apoptosis of the EC cells by directly suppressing TP53INP1 [23]. A high level of miR-106b was reported in EC and it enhanced the proliferation but inhibited apoptosis by suppressing p21 and Bim [24]. miR-204 was decreased in EC and further targeted FOXC1. Meanwhile, high expression of miR-204 in EC boosted the metastasis and infiltration of the EC cell HEC-1-A [25]. It can be seen that the detection of miRNA expressions in EC can help to evaluate the role of miRNAs. miR-641 has been found in various types of tumors acting as a tumor suppressor. For instance, Kong et al. found that miR-641 was dropped in lung cancer tissues and overexpression of miR-641 blocked the proliferation and induced apoptosis of lung cancer cells via sponging MDM2 [26]. Yao et al. manifested that upregulation of miR-641 deterred the proliferation of cervical cancer cells [27]. Hinske et al. found a low level of miR-641 in glioblastoma and it regulated the activation of AKT2 [15]. However, the possible mechanisms of miR-641 on EC remained unclarified. Here, we found that the miR-641 expression was low in the EC cells and its overexpression weakened proliferation and metastasis, reinforced apoptosis, and induced cell cycle arrest in the G1 phase. These results were consistent with previous research which verified that miR-641 acted as a tumor suppressor miRNA in EC.

miRNAs can promote or inhibit cancer progression by binding with their targets. Thus, the aim to study the mechanisms of miRNAs is to find their downstream targets [28, 29]. Because miRNA functioned by binding to 3'-UTR of target genes [30], AP1G1 was selected as a possible target of miR-641 via StarBase [31]. Furthermore, DLR assay proved that AP1G1 was sponged by miR-641. It has also been found that AP1G1 was highly expressed in several cancers and it was diminished in colon cancer tissues and cell lines, and silencing AP1G1 restored the role of HCP5 to slow down colon cancer progression [16]. Besides, the overexpression of AP1G1 reversed the promotive effect of lowly expressed MEG3 on the attack of liver cancer [17]. Moreover, AP1G1 was closely related to ASCT2-EGFR mediated with cetuximab and sensitization of head and neck squamous cell carcinoma cells [18]. Thus, our study found that AP1G1 was overexpressed in the EC cells, and overexpression of AP1G1 counteracted the functions of miR-641 on viability, proliferation, apoptosis, and metastasis of the EC cells.

RETRACTED

Taken together, we presented that the miR-641 expression was tarnished in the EC cells. The upregulation of miR-641 inhibited viability, proliferation, migration and invasion, accelerated apoptosis, and triggered cell cycle arrest in the G1 phase of the EC cells via targeting AP1G1. This study provides strong evidence that miR-641 might be an effective target for the treatment of EC.

## Figures and Tables

**Figure 1:** miR-641 is downregulated in the EC cells and upregulation of miR-641 inhibits viability and proliferation of the EC cells. (a) The expression level of miR-641 in the EC cells was detected by RT-qPCR assay. (b) The expression level of miR-641 in HEC-1A and HECCL-1 cells transfected with miR-641 mimic was evaluated by RT-qPCR assay. (c) The viability of HEC-1A and HECCL-1 cells transfected with miR-641 mimic was assessed by CCK-8 assay at indicated times. (d) The proliferation of HEC-1A and HECCL-1 cells transfected with miR-641 mimic was evaluated by colony formation assay. ^*∗*^*P* < 0.05, ^*∗∗*^*P* < 0.01, ^*∗∗∗*^*P* < 0.001 vs. miR-641 mimic NC.

**Figure 2:** Upregulation of miR-641 promotes apoptosis and induces G1 phase arrest of the EC cells. (a) The apoptotic rate of HEC-1A and HECCL-1 cells transfected with miR-641 mimic was determined by flow cytometry assay. (b) The cell cycle of HEC-1A and HECCL-1 cells transfected with miR-641 mimic was determined by flow cytometry assay. (c) The expression levels of proteins, including Cyclin D1, CDK2, and P21, were evaluated by western blot assay. ^*∗*^*P* < 0.05, ^*∗∗*^*P* < 0.01, ^*∗∗∗*^*P* < 0.001 vs. miR-641 mimic NC.

**Figure 3:** Upregulation of miR-641 inhibits migration and invasion of the EC cells. (a) The migration of HEC-1A and HECCL-1 cells transfected with miR-641 mimic was determined by wound healing assay. (b) The migration and invasion of HEC-1A and HECCL-1 cells transfected with miR-641 mimic were determined by the transwell migration and invasion assays. (c) The expression levels of proteins, including Cox-2, MMP-2, and MMP-9, were evaluated by western blot assay. ^*∗*^*P* < 0.05, ^*∗∗*^*P* < 0.01, ^*∗∗∗*^*P* < 0.001 vs. miR-641 mimic NC.

**Figure 4:** AP1G1 is a direct target of miR-641 in the EC cells. (a) The target gene of miR-641 was predicted with StarBase. (b) Dual luciferase reporter analysis was employed to validate the coactions between AP1G1 and miR-641. (c) The mRNA expression of AP1G1 in HEC-1A and HECCL-1 cells transfected with miR-641 mimic was evaluated by RT-qPCR assay. (d) The protein expression of AP1G1 in HEC-1A and HECCL-1 cells transfected with miR-641 mimic was evaluated by western blot assay. ^*∗*^*P* < 0.05, ^*∗∗*^*P* < 0.01, ^*∗∗∗*^*P* < 0.001 vs. miR-641 mimic NC.

**Figure 5:** AP1G1 mediates the effect of miR-641 on the EC cells. (a) The expression of AP1G1 in HEC-1A and HECCL-1 cells infected with Lv-AP1G1 was evaluated by RT-qPCR assay. (b) The viability of HEC-1A and HECCL-1 cells infected with Lv-AP1G1 was assessed by CCK-8 assay at indicated times. (c) The proliferation of HEC-1A and HECCL-1 cells infected with Lv-AP1G1 was evaluated by colony formation assay. (d) The apoptotic rate of HEC-1A and HECCL-1 cells infected with Lv-AP1G1 was determined by flow cytometry assay. (e) The migration of HEC-1A and HECCL-1 cells infected with Lv-AP1G1 was determined by the transwell migration assay. ^*∗*^*P* < 0.05, ^*∗∗*^*P* < 0.01, ^*∗∗∗*^*P* < 0.001 vs. NC mimic + Lv-NC. ^#^*P* < 0.05, ^##^*P* < 0.01, ^###^*P* < 0.001 vs. miR-641 mimic + Lv-NC.

RETRACTED

## Data Availability

The datasets generated/analyzed during the current study are available.
